# Effects of Neuromuscular Electrical Stimulation Combined with Repetitive Transcranial Magnetic Stimulation on Upper Limb Motor Function Rehabilitation in Stroke Patients with Hemiplegia

**DOI:** 10.1155/2022/9455428

**Published:** 2022-01-04

**Authors:** Junqiu Du, Shouyong Wang, Yun Cheng, Jiang Xu, Xuejing Li, Yimin Gan, Liying Zhang, Song Zhang, Xiaorui Cui

**Affiliations:** ^1^Department of Rehabilitation Medicine, Huai'an Second People's Hospital (The Affiliated Huai'an Hospital of Xuzhou Medical University), Huai'an, Jiangsu 223002, China; ^2^Department of Neurology, Huai'an NO.3 People's Hospital, Huai'an, Jiangsu 223002, China; ^3^Department of Rehabilitation Medicine, Huai'an NO.3 People's Hospital, Huai'an, Jiangsu 223002, China; ^4^Department of Rehabilitation Medicine, Lianshui County People's Hospital (Affiliated Hospital of Kangda College, Nanjing Medical University), Huai'an, Jiangsu 223400, China

## Abstract

**Objective:**

To investigate the effect of neuromuscular electrical stimulation (NMES) combined with repetitive transcranial magnetic stimulation (rTMS) on upper limb motor dysfunction in stroke patients with hemiplegia.

**Methods:**

A total of 240 stroke patients with hemiplegia who met the inclusion criteria were selected and randomly divided into 4 groups (60 cases in each group): control group, NMES group, rTMS group, and NMES + rTMS group. Before treatment and 4 weeks after treatment, we evaluated and compared the results including Fugl-Meyer assessment of upper extremity (FMA-UE) motor function, modified Barthel index (MBI), modified Ashworth scale (MAS), and motor nerve electrophysiological results among the 4 groups.

**Results:**

Before treatment, there was no significant difference in the scores of FMA-UE, MBI, MAS, and motor nerve electrophysiological indexes among the four groups, with comparability. Compared with those before treatment, the scores of the four groups were significantly increased and improved after treatment. And the score of the NMES + rTMS group was notably higher than those in the other three groups.

**Conclusion:**

NMES combined with rTMS can conspicuously improve the upper extremity motor function and activities of daily life of stroke patients with hemiplegia, which is worthy of clinical application and promotion.

## 1. Introduction

Stroke is an acute, focal, or diffuse injury to the central nervous system and characterized by high morbidity, high recurrence rate, high disability rate, and high mortality [1, 2]. According to the World Health Organization (WHO), approximately 70% of stroke survivors suffer from motor dysfunction [3]. Among them, hemiplegia is a common complication of stroke survivors [4, 5]. It is featured by abnormal motor function of the face and one side of the extremity, which is manifested by reduced resistance to passive movements and weakened or absent stretch reflex [6]. Hemiplegia usually occurs in the early stages of stroke and can lead to lifelong disability if not treated timely or properly.

In the past two decades, with the deepening of stroke research, more and more investigators have found that despite the central nervous system is damaged, there is still a possibility the function of the damaged nerve can be restored [7]. Recent studies have shown that plastic changes in the central nervous system may be closely related to poststroke rehabilitation [8, 9]. As for the methods of rehabilitation treatment, quite a few domestic and foreign literatures have reported that the group training treatment model can achieve satisfactory results, but the effect is relatively slow. Neuromuscular electrical stimulation (NMES) has been applied to the treatment of stroke patients since the last century [10]. The peak current of NMES with a specific waveform can maximize the number of responsive motor units and the rate at which they are generated, resulting in tonic contraction and powerful force [11]. The application of NMES can not only improve muscle strength but also reduce the spasm of muscles by inducing relaxation or mutual inhibition by maximum contraction [12]. Bakhtiary and Fatemy [13] found that NMES observably improved the muscle strength of anterior tibial muscle and ankle dorsiflexion muscle and the static spasm of plantar flexor. Barth et al. [14] also suggested that the application of electromyographic- (EMG-) triggered NMES to the anterior tibial muscle five days per week for 4 weeks in patients with chronic stroke could improve the range of motion of ankle dorsiflexion, balance, and gait. You et al. [15] emphasized the potential efficacy of NMES in the treatment of foot drop and showed that NMES has a beneficial help in the recovery of spasm after stroke.

Transcranial magnetic stimulation (TMS) as a new technique and means to promote the recovery of motor function after stroke has been extensively concerned and studied. It uses pulsed magnetic field to produce an induced current, which activates neurons in the central nervous system, resulting in changes in electrophysiology and function [16]. Repetitive transcranial magnetic stimulation (rTMS) is a series of TMS pulses that continuously act on the local brain. As a noninvasive neurophysiological stimulation technique, it has the characteristics of painless, noninvasive, nonattenuation, simple local operation, safe and effective, etc., which can effectively improve the efficacy of training and promote the recovery of upper limb dysfunction in stroke patients [17, 18]. In recent years, studies have combined NMES and rTMS for the treatment of upper extremity motor impairment after stroke. A randomized controlled trial by Tosun et al. showed that rTMS with or without NMES promoted motor recovery of the upper extremity in stroke patients [19]. Etoh et al. [20] demonstrated that rTMS partially promoted the improvement of hand function in stroke patients with hemiplegia. However, due to the small sample size in the current study, the effectiveness of NMES combined with rTMS treatment in upper limb motor rehabilitation in stroke is not clear. Therefore, this study further increased the experimental sample size to intervene in patients with hemiplegic upper limb dysfunction after stroke by NMES combined with rTMS to clarify the clinical efficacy of this combined treatment modality in upper limb dysfunction after stroke.

## 2. Materials and Methods

### 2.1. General Information

We collected 240 stroke patients with hemiplegia admitted to our hospital from June 2017 to March 2020, and the diagnosis was in accordance with the diagnostic criteria established by the Global Academic Conference on Cerebrovascular Disease. According to the treatment plan, the patients were randomly divided into four groups (60 cases in each group): (1) control group, only routine treatment; (2) NMES group, NMES on the basis of routine treatment; (3) rTMS group, rTMS on the basis of routine treatment; and (4) NMES+rTMS group, NMES combined with rTMS at the same time on the basis of routine treatment. This was an assessor-blinded randomized controlled study. This study protocol has been reviewed by the medical ethics committee of our hospital, and all subjects have voluntarily signed the informed consent form.

The inclusion criteria are as follows: (1) all patients were diagnosed with stroke by CT or MRI; (2) all were the first-episode; (3) with typically unilateral limb hemiplegia, and there is pain in the affected shoulder, affecting the upper limb motor function; (4) no serious disturbance of consciousness and communication disorders; (5) the course of the disease is less than 3 months; (6) Brunnstrom stage of the upper limb ≥ II; and (7) all the patients are adults (age > 18 years).

The exclusion criteria are as follows: (1) suffering from brain diseases such as Parkinson's disease and brain tumor; (2) having a cardiac pacemaker, implanted defibrillator, or other implantable devices in the body; (3) having a history of epilepsy and family history of epilepsy; (4) severe hepatic and renal insufficiency and severe infection; (5) obvious cognitive impairment, unable to understand and cooperate with instructions; and (6) patients with severe spasm or contracture of the upper limb.

### 2.2. Treatment Method

The participants were divided into four groups, and the corresponding treatment was performed according to the frequency of once a day, 5 days a week, and 4 consecutive weeks. The details are as follows: (1) control group: only carrying on rehabilitation training, including physiotherapy and task-oriented occupational therapy, mainly with Bobath and Rood techniques. Including limb position, antispasm training, joint range of motion maintenance training, upper limb movement control training, key muscle group muscle strength training, deep and shallow sensation training, daily living ability training, and each treatment lasted for 45 min. (2) NMES group: On the basis of rehabilitation training, RH-ZP-D surface neuromuscular stimulation therapy instrument (Henan Ruihe Medical Equipment Co., Ltd.) was used for NMES. Surface electrodes were placed on the extensor carpi and extensor digitorum communis muscles. The bidirectional symmetric TENS waveform and pulse phase duration were 200 *μ*s, and the frequency was 50 Hz, and current intensity was adjusted until significant muscle contraction occurred, and each treatment lasted 30 min; (3) rTMS group: on the basis of rehabilitation training, CCY-I TMS with a coil (Wuhan Eruid Medical equipment New Technology Co., Ltd.) was used to stimulate the primary motor cortex (M1) of the intact cerebral cortex. The stimulation frequency was 1 Hz, and the stimulation intensity was 90% resting motor threshold (RMT). A total of 1200 pulses with a duration of 20 min. RMT was determined by observing the maximum flexion of the contralateral index finger achieved in more than 5 out of 10 single-pulse stimuli. The site of stimulation was the site where the RMT was determined [19]. (4) NMES+rTMS group: the patients were treated with NMES and rTMS at the same time on the basis of routine rehabilitation training.

### 2.3. Observation Indicators

1. Modified Barthel Index (MBI) scale was used to assess the patient's activities of daily living, including 10 items such as eating, bathing, dressing, and modifying. The scoring standard is as follows: 100 were completely independent; 95-75 were classified as mild dysfunction; 70-50 were classified as moderate dysfunction; 50-25 were classified as severe dysfunction and obvious life dependence; ≤20 is totally dependent in life
2. The upper extremity portion of the Fugl-Meyer motor assessment (FMA-UE) was used to assess the improvement of upper limb and hand function in patients, including 33 items, each of which was 0-2 points for a total of 3 levels. The specific scoring criteria were as follows: 0 point, unable to complete; 1 point, partially complete; 2 points, all complete. The total score was 66 points, and the higher the score, the better the motor function of the upper limb
3. Modified Ashworth Scale (MAS) was used to evaluate the muscle tension of the elbow, wrist, and finger, which was divided into 1-4 grades, and the higher the level, the higher the muscle tension was suggested
4. Changes in motor evoked potentials (MEPs) induced by TMS were detected by using different coil orientations [21]. Central motor conduction time (CMCT) was measured with reference to the previous method [22]. MEPs and CMCT were mainly used to observe the physiological changes of movement in poststroke hemiplegic patients

### 2.4. Statistical Analysis

The statistical software was preformed using the SPSS22.0. When the measurement data were normally distributed, the results were represented as mean ± standard deviation (SD). Analysis of variance was used for the comparison among multiple groups, and the paired *t*-test was used for the intragroup comparison before and after the treatment. If the data did not meet normal distribution, the results were expressed as median (quartile). Wallkalis *H* test was used for comparison among multiple groups. Mann–Whitney *U* test was used for comparison between two groups. Wilcoxon signed-rank test was used for comparison pre- and postinterventions in the intragroup. Enumeration data were expressed as *n* (%), and Chi-square test was used for comparison. *P* < 0.05 was considered statistically significant.

## 3. Results

### 3.1. Clinical General Data

General clinical information was collected for all subjects. As shown in Table 1, there were no significant differences in patient gender, age, body mass index (BMI), disease course, dominant hand, stroke type, hemiplegic direction, and Brunstrom stage among the groups (*P* < 0.05).

### 3.2. NMES and rTMS Improve Modified Barthel Index in Patients after Treatment

The patients' activities of daily living were evaluated by MBI. The results showed that there was no significant difference in MBI among patients in the control group, NMES group, rTMS group, and NMES+rTMS group before treatment (Table 2, *P* > 0.05), which were comparability. MBI was significantly increased after treatment in all four groups compared with that before treatment. Among them, patients in the NMES + rTMS group (71.30 ± 5.69) had a significantly higher MBI than the other groups. MBI in the NMES group (67.98 ± 6.59) and rTMS group (68.35 ± 5.42) were higher than the control group (63.87 ± 7.16) (Table 2, *P* < 0.05), and there was no significant difference between NMES and rTMS group (*P* > 0.05).

### 3.3. NMES and rTMS Improve Fugl-Meyer Assessment of Upper Extremity in Patient Treatment

The improvement of upper limb (UL) function was assessed by FMA-UE. The scoring results showed that no significant difference in UL-FMA among the four groups before treatment (Table 3, *P* > 0.05). Compared with the pretreatment period, UL-FMA was considerably higher after treatment in all four groups. The UL-FMA of patients in the NMES + rTMS group (33.80 ± 4.16) was significantly high than that in the other three groups, and the UL-FMA of patients in the NMES group (30.83 ± 5.60) and rTMS group (31.77 ± 5.83) was obviously increased than that in the control group (27.27 ± 4.40) (Table 3, *P* < 0.05), while there was no significant difference between the NMES group and the rTMS group.

### 3.4. NMES and rTMS Improve Modified Ashworth Scale in Patients after Treatment

The muscle tension of the elbow, wrist, and finger was evaluated by MAS. As shown in the results in Table 4, there were no significant differences in MAS of the elbow, wrist, and finger in patients in the control, NMES, rTMS, and NMES+rTMS group before treatment (Table 4, *P* > 0.05). In comparison with those before treatment, the MAS of the elbow, wrist, and finger were observably raised in the NMES + rTMS group after treatment. Only the MAS of the finger was significantly increased in the NMES group and rTMS group, and the MAS of the elbow only was notably improved in the control group (Table 4, *P* < 0.05).

### 3.5. NMES and rTMS Improve Motor Nerve Electrophysiology in Patients after Treatment

According to the data of motor nerve electrophysiological index, there was no significant difference in CMCT and MEP among the four groups before treatment (Table 5, *P* > 0.05). Contrasted with that before treatment, the CMCT and MEP of patients in the four groups were significantly reduced after treatment. The CMCT and MEP of patients in the NMES + rTMS group (CMCT, 10.03 ± 1.81; MEP, 20.17 ± 3.46) were notably decreased than the other three groups, and the CMCT and MEP of patients in the NMES group (CMCT, 10.85 ± 1.53; MEP, 21.62 ± 3.15) and the rTMS group (CMCT, 10.73 ± 1.56; MEP, 21.43 ± 3.09) were significantly shorten than those in the control group (CMCT, 11.60 ± 1.29; MEP, 23.05 ± 3.40) (Table 5, *P* < 0.05).

## 4. Discussion

In recent years, stroke has shown the characteristics of younger age and high recurrence rate [23], which has seriously affected the quality of life of patients and caused a huge burden to families and society. Due to the projection area of the hand and upper limb in the cerebral cortex is relatively large, once damaged, its function recovery is very difficult. How to recover the upper limb, especially the hand function, is still the focus and difficulty of stroke rehabilitation treatment at present [24]. Studies have shown that the motor cortex of the affected hemisphere has diminished inhibitory effects on the motor cortex of the intact hemisphere after stroke [25]. Therefore, in order to restore the function of the upper limbs and hands of the patients, on the one hand, it can increase the excitability of the damaged brain areas; on the other hand, it is necessary to improve the mutual inhibition between the two hemispheres to promote brain balance.

Numerous studies have confirmed that NMES has a prominent effect on limb rehabilitation in stroke patients. Some studies have shown that electrical stimulation therapy plays a positive role in relieving shoulder pain and improving muscle function in patients with stroke [26–28]. Its main advantage lies in the regulation of brain function in a noninvasive way, and its strong spatial localization ability, which provide a broad room for the treatment of different brain functional areas [29]. Yang et al. [30] discovered that NMES of ankle dorsiflexor can effectively improve gait performance and ankle control in patients with chronic stroke. Since the first TMS was successfully developed and MEP was elicited in 1985 by British scientist Barker et al., rTMS has been developed for nearly 30 years and has received extensive attention and research [31]. Researches have shown that rTMS can improve the motor function of stroke patients, such as Beynel et al. were used 1 Hz rTMS to act on the upper limb projection area of the unaffected side of the brain M1 area. The results suggest that rTMS can reduce upper limb spasm in stroke patients [32]. In recent years, with the progress of functional imaging, molecular biology and physical factor therapy techniques, and other related disciplines, the study of brain function after stroke and the recovery of upper limb and hand dysfunction has been increasingly refined [30]. And with the further development of clinical combined therapy, a plenty of studies have shown that combined therapy shows a better effect, such as Balderston et al. using rTMS combined with rehabilitation training to treat cerebral infarction patients with hemiplegic. The results show that rTMS combined with rehabilitation therapy can effectively improve the motor function of hemiplegic patients with cerebral infarction [33]. For this purpose, in this study, on the basis of rehabilitation training, NMES combined with rTMS were used to explore the effect of the combination of the two on upper limb dysfunction in stroke patients with hemiplegia. The results indicated that compared with single application, the combination of the two could significantly improve the activities of daily living, upper extremity motor function, muscle tension, and motor nerve function of patients. To sum up, NMES combined with rTMS not only improves the efficacy of upper limb function in stroke patients with hemiplegia but also provides a new painless and noninvasive treatment technique for neurological rehabilitation of poststroke, especially upper limb motor dysfunction. At the same time, this study suggests that the combination of the two is helpful to improve the efficacy of rehabilitation training, providing theoretical and experimental basis for the rehabilitation of upper limb motor function diseases in stroke patients with hemiplegia, and it is recommended to be widely used.

However, due to the large number of parameters and complex mechanism of NMES combined with rTMS, different parameter combinations will produce different effects, which brings difficulties to the development of the best treatment plan, so this study still has many shortcomings. It is necessary to study and solve the influences of parameters such as the number of pulses of different stimuli, duration, and interval time and the total pulse number of each treatment on the therapeutic effect and long-term effect, so as to formulate the best treatment plan for each patient and obtain the best curative effect and to maximize the benefit of NMES combined with rTMS.

## Figures and Tables

**Table 1:** Comparison of clinical characteristics of patients in each group.

Characteristics	Control group (*n* = 60)	NMES group (*n* = 60)	rTMS group (*n* = 60)	NMES+rTMS group (*n* = 60)	*X* ^2^/*F*	*P*
Age (year)	57.2 ± 8.95	58.77 ± 8.39	59.05 ± 8.9	58.22 ± 9.98	0.485	0.693
Gender (%)					1.735	0.629
Male	34 (56.7)	28 (46.7)	33 (55)	29 (48.3)		
Female	26 (43.3)	32 (53.3)	27 (45)	31 (51.7)		
BMI (kg/m^2^)	23.87 ± 3.09	23.91 ± 3.37	24.15 ± 3.3	23.8 ± 3.43	0.129	0.943
Disease course (month)	47.02 ± 14.21	50.25 ± 11.78	45.95 ± 12.73	47.7 ± 12.37	1.224	0.302
Dominant hand (%)					2.459	0.483
Left	6 (10)	3 (5)	2 (3.3)	4 (6.7)		
Right	54 (90)	57 (95)	58 (96.7)	56 (93.3)		
Stroke type (%)					3.055	0.383
ICH	14 (23.3)	20 (33.3)	12 (20)	15 (25)		
IS	46 (76.7)	40 (66.7)	48 (80)	45 (75)		
Hemiplegic direction (%)					1.765	0.623
Left	34 (56.7)	35 (58.3)	37 (61.7)	30 (50)		
Right	26 (43.3)	25 (41.7)	23 (38.3)	30 (50)		
Brunstrom stage (%)					2.705	0.997
II stage	23 (38.3)	21 (35)	21 (35)	20 (33.3)		
III stage	15 (25)	16 (26.7)	18 (30)	21 (35)		
IV stage	10 (16.7)	10 (16.7)	8 (13.3)	8 (13.3)		
V stage	8 (13.3)	9 (15)	8 (13.3)	6 (10.0)		
VI stage	4 (6.7)	4 (6.7)	5 (8.3)	5 (8.3)		

**Table 2:** Comparison of MBI in different groups of patients before and after treatment.

Group	Cases	MBI before treatment	MBI after treatment	*t*	*P*
Control group	60	55.37 ± 5.39	63.87 ± 7.16	6.996	0.001
NMES group	60	56.20 ± 5.09	67.98 ± 6.59^∗^^a^	11.275	0.001
rTMS group	60	55.88 ± 6.61	68.35 ± 5.42^∗^^a^	10.265	0.001
NMES+rTMS group	60	56.08 ± 4.76	71.30 ± 5.69^∗^^abc^	16.059	0.001
*F*		0.269	14.33		
*P*		0.848	0.000		

^∗^ *P* < 0.05 vs. before treatment; ^a^*P* < 0.05 vs. control group; ^b^*P* < 0.05 vs. NMES group; ^c^*P* < 0.05 vs. rTMS group.

**Table 3:** Comparison of FMA-UE in different groups of patients before and after treatment.

Group	Cases	FMAUE before treatment	FMAUE after treatment	*t*	*P*
Control group	60	24.30 ± 4.15	27.27 ± 4.40	3.821	0.001
NMES group	60	23.27 ± 3.28	30.83 ± 5.60^∗^^a^	8.771	0.001
rTMS group	60	23.40 ± 4.04	31.77 ± 5.83^∗^^a^	9.032	0.001
NMES+rTMS group	60	24.35 ± 4.18	33.80 ± 4.16^∗^^abc^	12.44	0.001
*F*		1.287	17.529		
*P*		0.280	0.000		

^∗^ *P* < 0.05 vs. before treatment; ^a^*P* < 0.05 vs. control group; ^b^*P* < 0.05 vs. NMES group; ^c^*P* < 0.05 vs. rTMS group.

**Table 4:** Comparison of MAS in different groups of patients before and after treatment.

Group	Cases	Elbow		Wrist		Finger	
		Before treatment	After treatment	Before treatment	After treatment	Before treatment	After treatment
Control group	60	2 (2-2)	2 (2-3)	2 (1-2)	2 (2-3)	1.5 (1-2)	2 (2-3)
NMES group	60	2 (2-2)	3 (2-3)^∗^^a^	1.5 (1-2)	2.5 (2-3)^∗^^a^	2 (1-2)	3 (2-3)^∗^^a^
rTMS group	60	2 (2-2)	3 (3-3.5)^∗^^a^	2 (1-2)	3 (2-3)^∗^^a^	2 (1-2)	3 (2-3)^∗^^a^
NMES+rTMS group	60	2 (2-2)	3 (3-4)^∗^^abc^	2 (1-2)	3 (2.5-3)^∗^^abc^	2 (1-2)	3 (2-4)^∗^^abc^
*H*		1.543	32.082	2.477	32.879	1.483	29.294
*P*		0.672	0.001	0.479	0.001	0.686	0.001

^∗^ *P* < 0.05 vs. before treatment; ^a^*P* < 0.05 vs. control group; ^b^*P* < 0.05 vs. NMES group; ^c^*P* < 0.05 vs. rTMS group.

**Table 5:** Comparison of motor nerve electrophysiology in different groups of patients before and after treatment.

Group	Cases	MEP		CMCT	
		MEP before treatment	MEP after treatment	CMCT before treatment	CMCT after treatment
Control group	60	27.05 ± 3.35	23.05 ± 3.40^∗^	13.10 ± 1.35	11.60 ± 1.29^∗^
NMES group	60	26.67 ± 2.52	21.62 ± 3.15^∗^^a^	12.97 ± 1.30	10.85 ± 1.53^∗^^a^
rTMS group	60	26.50 ± 3.39	21.43 ± 3.09^∗^^a^	12.87 ± 1.57	10.73 ± 1.56^∗^^a^
NMES+rTMS group	60	26.63 ± 3.40	20.17 ± 3.46^∗^^abc^	13.13 ± 1.28	10.03 ± 1.81^∗^^abc^

^∗^ *P* < 0.05 vs. before treatment; ^a^*P* < 0.05 vs. control group; ^b^*P* < 0.05 vs. NMES group; ^c^*P* < 0.05 vs. rTMS group.

## Data Availability

The data used to support the findings of this study are available from the corresponding author upon request.
